# *Spondias purpurea* L. Bark Extract Protects against Oxidative Stress and Reduces Hypercholesterolemia in Mice Fed High-Fat Diet

This article has been retracted.

**DOI:** 10.1155/2022/3046483

**Published:** 2022-03-31

**Authors:** Kátia A. Antunes, Tamaeh Monteiro-Alfredo, Janielle S. M. Cunha, Priscila P. T. Espindola, Alex S. Oliveira, Caio F. Ramalho de Oliveira, José Tarcísio G. de Carvalho, Nelson L. C. Domingues, Denise B. Silva, Silvia C. F. Olinto, Edson L. dos Santos, Kely de Picoli Souza

**Affiliations:** ^1^Research Group on Biotechnology and Bioprospecting Applied to Metabolism, Federal University of Grande Dourados, Dourados, Brazil; ^2^Federal University of Amapá, Amapá, Brazil; ^3^Laboratory of Natural Products and Mass Spectrometry, Federal University of Mato Grosso Do Sul, Campo Grande, Brazil

## Abstract

Oxidative stress plays a key role in the initiation and progression of metabolic diseases, including obesity. Preventing the accumulation of reactive oxygen species and oxidative damage to macromolecules is a beneficial strategy for reducing comorbidities associated with obesity. Fruits from the *Spondias* genus are known for their antioxidant activity, but they are not available year-round due to their seasonality. In this context, we investigated the antioxidant activity and identified the chemical constituents of the aqueous extract of the stem bark of *Spondias purpurea* L. (EBSp). Additionally, we evaluated the effect of EBSp consumption on metabolic parameters in mice with obesity induced by a high-fat diet. Chemical analyses revealed 19 annotated compounds from EBSp, including flavan-3-ols, proanthocyanidins, methoxylated coumarin, and gallic and ellagic acids, besides other phenolic compounds. In vitro, EBSp showed antioxidant activity through the scavenging of the free radicals and the protection of macromolecules against oxidative damage. Cellular assays revealed that EBSp reduced the levels of malondialdehyde produced by erythrocytes exposed to the oxidizing agent AAPH. Flow cytometry studies showed that EBSp reduced reactive oxygen species levels in human peripheral blood mononuclear cells treated with hydrogen peroxide. Obese mice treated with EBSp (400 mg.kg^−1^) for 60 days showed reduced levels of malondialdehyde in the heart, liver, kidneys, and nervous system. The total cholesterol levels in mice treated with EBSp reached levels similar to those after treatment with the drug simvastatin. Together, the results show that the combination of the different phenolic compounds in *S. purpurea* L. bark promotes antioxidant effects in vitro and in vivo, resulting in cytoprotection in the context of oxidative stress associated with obesity and a reduction in hypercholesterolemia. From a clinical perspective, the reduction in oxidative stress in obese individuals contributes to the reduction in the emergence of comorbidities associated with this metabolic syndrome.

## 1. Introduction

Physiological cellular processes continuously produce reactive species (REs) in the body. However, exogenous stressors, such as high-fat diets, contribute to the increase in these levels [1]. When the level of REs exceeds the antioxidant capacity of the organism, damage to macromolecules (proteins, lipids, and nucleic acids) is observed. The accumulation of these deleterious effects triggers the development of several diseases, including obesity, dyslipidemia, atherosclerosis, hypertension, and vascular endothelial dysfunction [1–4].

To protect an organism from deleterious oxidative effects, the endogenous antioxidant system—including enzymatic and nonenzymatic processes—can neutralize oxidative damage [5, 6]. To ensure that REs are completely neutralized, the intake of exogenous antioxidants is necessary [7]. In this sense, plants are an important source of antioxidant compounds, a feature attributed to several chemical constituents that act individually or synergistically [8].

Plant species from *Spondias* genus (Anacardiacea) have several phenolic compounds that are effective in reducing lipid peroxidation and protein oxidation in vitro [9, 10]. *Spondias purpurea* is a species native to Mexico but widely distributed in Central and South America, including Brazil. Although there are few studies on *S. purpurea*, the antioxidant activity of leaf and fruit extracts has been described [10, 11], in addition to antiulcerogenic [11] and antiglycation [12] properties. Nevertheless, there are no studies on the chemical constituents present in the stem bark of *S. purpurea*, nor their pharmacological properties. Additionally, since the popular use of *S. purpurea* involves the decoction of the stem bark for the treatment of conditions such as diarrhea and dysentery, we investigated the chemical composition of the aqueous extract of the stem bark of *S. purpurea* (EBSp) and evaluated the antioxidant properties of EBSp *in vitro*. In addition, we evaluated the pharmacological properties of EBSp *in vivo* using a mouse model of obesity induced by a high-fat diet, in which anthropometric and biochemical parameters were assessed.

## 2. Materials and Methods

### 2.1. Reagents

Electrophoresis, DCFH (2′,7′-dichlorofluorescin diacetate), Folin-Ciocalteu, DPPH (2,2-diphenyl-1-picrylhydrazyl), ABTS (2,2′-Azinobis-(3-ethylbenzothiazoline-6-sulfonic acid)), and AAPH (2,2′-Azobis(2-methylpropionamidine) dihydrochloride) reagents were acquired from Sigma-Aldrich (São Paulo, Brazil). Catechin, quercetin, tiobarbituric acid (TBA), sulfuric acid, sodium carbonate, aluminum chloride, hexane, sodium hydroxide, methanol, and hydrogen peroxide were purchased from Merck (São Paulo, Brazil). Ascorbic acid and gallic acid of analytical degree were acquired from Dinâmica (São Paulo, Brazil).

### 2.2. Preparation of Aqueous Extract of *Spondias purpurea* L. Stem Bark (EBSp)

The *S. purpurea* L. stem bark was collected in Itaporã, Mato Grosso do Sul, Brazil (S 21° 54′ 33.3^″^ and W 054° 42′ 04.9^″^), dried in an air circulation oven at 45 ± 5°C and ground in a Willey-knife mill. An exsiccate of the species was deposited at the Herbarium of the Federal University of Grande Dourados, Mato Grosso do Sul, Brazil, under voucher 5461. The aqueous extract was prepared by decoction of *S. purpurea* bark in distilled water at a ratio of 1 : 200 (*w*/*v*) for 1 h. Then, the extract was filtered, freeze-dried, and stored at -20°C, sheltered from light.

### 2.3. Chemical Analyses by Liquid Chromatography-Diode Array Detection-Mass Spectrometry (LC-DAD-MS)

The analysis of EBSp was performed in a UFLC chromatography Shimadzu Proeminence system coupled to a diode array detector and a mass spectrometer MicrOTOF-Q III (Bruker Daltonics), which is provided with an electrospray ionization source and analyzers quadrupole and time-of-flight. For the analyses, a Kinetex C18 chromatographic column (Phenomenex, 2.6 *μ*m, 100 Å, 150 × 2.1 mm) was used. The flow rate was 0.3 mL.min^−1^ and an injection volume was 8 *μ*L. The mobile phase was acetonitrile (B) and ultrapure water (A) with 0.1% formic acid (*v*/*v*). The chromatographic separation was performed by gradient elution profile (0-2 min -3% B, 2-25 min from 3 to 25% B, 25-40 min from 25 to 80% B, and 40-43 min -80% B) at 50°C. For the MS analyses, nitrogen is applied as nebulization gas (4 bar) and drying gas (9 L.min^−1^), applying the capillary voltage 3,500 kV. EBSp was analyzed by positive and negative ion mode.

### 2.4. Antioxidant Activity

#### 2.4.1. Free Radical ABTS and DPPH Scavenging

The antioxidant activity of EBSp was evaluated using the methods of ABTS and DPPH. The ABTS free radical scavenging capacity was determined using the method described by Rufino et al. (2010). An ABTS solution was prepared from an oxidation reaction that occurs between potassium persulfate (2.45 mM) and ABTS (7 mM), from 12 to 16 h before the assay. The assay was performed at room temperature. In a glass tube, 20 *μ*L of EBSp at different concentrations (1-2,000 *μ*g.mL^−1^) were mixed with 1,980 *μ*L of ABTS solution. The samples were incubated for 6 min, sheltered from light, and absorbance at 734 nm determined in a spectrophotometer (PG Instruments Limited, Leicestershire, United Kingdom). The percentage of ABTS scavenging was determined according to

(1) $$\begin{array}{c} \text{ABTS inhibition}\left(\%\right)=1-\left(\frac{\text{Abs sample}}{\text{Abs control}}\right)\times 100. \end{array}$$

The scavenging of DPPH free radical was determined according to Gupta & Gupta (2011). A volume of 200 *μ*L of ECPS in different concentrations (1-2,000 *μ*g.mL^−1^) were mixed to 1,800 *μ*L of the DPPH radical solution (0.11 mM, 80% ethanol), following incubation for 30 min, protected from light, and read at 517 nm. The percentage of DPPH inhibition was calculated according to:

(2) $$\begin{array}{c} \text{DPPH inhibition }\left(\%\right)=1-\left(\frac{\text{Abs sample}}{\text{Abs control}}\right)\times 100. \end{array}$$

Both assays were carried out in triplicate and represent the result of three independent assays.

### 2.5. Protection of Proteins against Oxidation Induced by AAPH

To determine the antioxidant potential of EBSp against oxidation induced by AAPH, we used bovine serum albumin (BSA) as standard. In a 200 *μ*L microtube, 7 *μ*g of BSA were incubated for 30 min at 37°C with different concentrations of EBSp (5-1,000 *μ*g.mL^−1^, final concentration). After this period, an AAPH solution (75 mM, final concentration), was mixed with the samples, and a new incubation period for 60 min at 37°C was carried out. Subsequently, samples were mixed with sample buffer (20% SDS, glycerol, 0.5 M Tris-HCl, pH 6.8, and 0.1% bromophenol blue), heated for 3 min at 95°C and applied onto a 12% polyacrylamide gel electrophoresis containing SDS (12% SDS-PAGE). The gel was stained, distained, and digitized using Gel Doc™ EZ System (BioRad), and the Image Lab™ software was used to determine the band volume. The average of 4 gels were used to determine the protection conferred by EBSp against protein oxidation, represented by reduction of BSA band volumes in comparison with positive treatment (BSA + AAPH).

#### 2.5.1. Protection against DNA Fragmentation Induced by Hydrogen Peroxide

The assay of protection against DNA fragmentation was performed according to Kumar & Chattopadhyay (2007), with some modifications. A plasmidial DNA of 5,597 bp (4 *μ*L at 50 ng.*μ*L^−1^) was mixed with 4 *μ*L of EBSp (5-100 *μ*g.mL^−1^) and with 30% hydrogen peroxide. The samples were incubated in 302 nm transilluminator (UVT-312) at room temperature for 5 min. Then, the samples were subjected to electrophoresis on 2% agarose gel containing ethidium bromide (10 mg.mL^−1^). The gel was digitized using the Gel Doc ™ EZ System (BioRad) and analyzed using the Image Lab ™ software. The average of 4 gels were used to determine the protection conferred by EBSp against DNA fragmentation.

#### 2.5.2. Determination of Hemolytic Activity, Inhibition of Oxidative Hemolysis Induced by AAPH, and Measurement of Malondialdehyde Levels

The experimental procedure was performed following the approval of the Research Ethics Committee CEP/UFGD 053161/2019. The protective effect of the EBSp against oxidative hemolysis was assessed with AAPH induction.

The blood from an adult and healthy donor was washed three times in NaCl (0.9%) and used to prepare an erythrocyte suspension at 10% (*v*/*v*). A volume of 250 *μ*L of the erythrocyte suspension was incubated for 30 min at 37°C in the presence of 250 *μ*L ascorbic acid (AA) (5-100 *μ*g.mL^−1^) or EBSp (5-100 *μ*g.mL^−1^). Subsequently, 500 *μ*L of NaCl (0.9%) or AAPH (50 mM) was added in the samples to assess the level of hemolysis and the inhibition of oxidative hemolysis, respectively. The samples were kept at 37°C for 240 min with periodic stirring. Three independent assays were carried out in duplicate. The percentage of hemolysis was assessed by measuring the absorbance at 540 nm according to

(3) $$\begin{array}{c} \text{Hemolysis }\left(\%\right)=\left(\frac{\text{Abs sample}}{\text{Abs total hemolysis}}\right)\times 100. \end{array}$$

For lipid peroxidation assay, a similar experiment was carried out as described early. At the end of 240 min of incubation, the samples were centrifuged at 2,000 rpm, and 500 *μ*L of the supernatant was transferred for tubes containing 1 mL of thiobarbituric acid (TBA, 10 nmol.L^−1^). As positive control, 500 *μ*L of MDA solution (20 *μ*M) was mixed with 1 mL of TBA. The samples were incubated at 96°C for 45 min. Then, 4 mL of n-butyl alcohol was added to each sample and was centrifuged at 2,000 rpm. The absorbance of the supernatants was measured at 532 nm. Two independent experiments were carried out in duplicate. The MDA content in samples was estimated according to Equation (4), expressed in nmol.mL^−1^.

(4) $$\begin{array}{c} \text{MDA}=\text{Abs sample}\times \left(\frac{20\text{ x }220.32}{\text{Abs positive control}}\right). \end{array}$$

#### 2.5.3. Oxidative Stress Induced by Hydrogen Peroxide in Peripheral Blood Mononuclear Cells

Peripheral blood mononuclear cells (PBMC) were isolated using Ficoll-Paque (GE Healthcare) and transferred to 12-well plates at a density of 5 × 10^5^ cells per well. PBMC were incubated with 2,000 *μ*L of different concentrations of the EBSp (5-100 *μ*g.mL^−1^) at 37°C and 5% CO_2_ atmosphere. After 24 h, 15 *μ*L of hydrogen peroxide (H_2_O_2_) (10 mM) was added to the wells to induce oxidative stress during 30 min. Then, PBMC were washed with PBS and incubated 100 *μ*L of DCFH (10 mM) to determine the intracellular levels of ROS by flow cytometry, collecting 10,000 events in a BD Accuri C6 Plus cytometer (BD Biosciences). The ROS levels were determined by quantifying the mean fluorescence intensity (MFI) in FITC-A. Results were presented as an average of three experiments carried out in triplicate.

### 2.6. Animal Experimentation

#### 2.6.1. Ethics Committee

The study was carried out according to the ethical principles for animal experimentation, adopted by the National Council for Animal Experimentation Control (CONCEA) and approved by the Animal Use Ethics Committee (CEUA) of the Federal University of Grande Dourados, Brazil, under the protocol number 37/2018.

#### 2.6.2. Acute Toxicity

Female C57BL/6 mice (*n* = 15) with 22 g of body mass were acclimated in vivarium under standard conditions (22 ± 2°C, 50–60% RU, light/darkness cycle of 12/12 h) and fed with commercial diet and water *ad libitum*. Subsequently, the mice were divided into three experimental groups and received a single dose of treatment by gavage: (I) CT (water), (II) EBSp-2 (EBSp 2 g.kg^−1^), and (III) EBSp-5 (EBSp 5 g.kg^−1^). Food and water intake, body mass, piloerection, and mortality were monitored during 14 days. After the treatment period, the mice were fasted for 8 h, anesthetized, and euthanized. Organs (liver, kidneys, spleen, heart, lung, and nervous system) were collected, weighed separately, and analyzed macroscopically. Additionally, blood samples were collected for hematological determinations using the COBAS analyzer (Roche Diagnostics).

#### 2.6.3. Evaluation of Metabolic Parameters

*(1) Diets*. Both standard (AIN-93M) and high-fat (HF9 60) diets were purchased from *PragSoluções Biociências* (São Paulo, Brazil). The standard rodent diet possessed 377 kcal.100.g^−1^. The lipid content in the high fat diet (60% of lipids) conferred a total caloric value of 576 kcal.100.g^−1^.

*(2) Design and Experimental Procedures*. Male C57BL/6 mice (*n* = 32) were divided into two groups, mice fed with the standard diet (CT) (*n* = 8) and mice fed with the high-fat diet (HFD) (*n* = 24) for 120 days, until the obtainment of obese mice. Afterwards, the mice from HFD group were subdivided into 3 groups (*n* = 8), which were treated by gavage for 60 days, using (I) water (HFD-CT), (II) simvastatin 30 mg.kg^−1^ (HFD-Simv), or (III) EBSp 400 mg.kg^−1^ (HFD-EBSp).

*(3) Organs and Tissues*. At the end of the period of treatment, the mice were anesthetized with ketamine and xylazine (1 : 1), and euthanized. The deposits of brown adipose tissue (BAT) and white adipose tissue (WAT) (retroperitoneal, epididymal, mesenteric, and subcutaneous inguinal), gastrocnemius muscle, eye, nervous system, pancreas, kidneys, spleen liver, heart, and duodenum were removed and weighed individually. Blood samples were collected from the aortic artery, and biochemical parameters (glycemia, total cholesterol, triglycerides, aspartate aminotransferase (AST), and alanine aminotransferase (ALT)) were determined by a semiautomatic biochemical analyzer (LABQUEST, Bioplus, Barueri, São Paulo, Brazil).

*(4) MDA Dosage in Organs*. The MDA content in organs was determined according to Cunha et al. (2018). Organ samples (eyes, heart, kidneys, liver, and nervous system) were homogenized with 1.1% KCl and centrifuged at 3,000 rpm for 10 min. Then, 500 *μ*L of tissue supernatant or 500 *μ*L of MDA standard (20 *μ*M) was added to 1 mL TCA (10%) and 1 mL of TBA (10 nmol.mL^−1^), followed by incubation at 96°C for 45 min. Samples were cooled for 15 min in an ice bath, followed by the addition of 3 mL of n-butyl alcohol and centrifugation at 3,000 rpm for 5 min. The absorbance was measured at 532 nm in a UV/VIS spectrophotometer model T70 (PG Instruments, Leicestershire, UK). The MDA content was expressed as nmol.mL^−1^, according to Equation (4).

### 2.7. Statistical Analysis

Data were expressed as mean ± standard error of the mean (SEM) and subjected to unidirectional analysis of variance (ANOVA) followed by Student Newman Keuls posttest. Results were considered significant when *P* < 0.05. Statistical analyses were performed with the statistical software GraphPad Prism 5.0.

## 3. Results

### 3.1. Chemical Compounds in EBSp

The LC-DAD-MS analyses (Figure S1, supplementary material) revealed 19 compounds, which were annotated based on their spectral data (UV, MS, and MS/MS) compared with literature data (Table 1). The molecular formulae were determined by accurate mass measurements considering an error and sigma up to 8 ppm and 20, respectively.

Compounds **1**, **2**, and **3** did not exhibit UV absorption and had the following molecular formulas, respectively: C_12_H_22_O_11_, C_6_H_8_O_8_, and C_6_H_8_O_7_ (Table 1). In addition, **1** and **2** showed losses of a hexosyl and a water molecule, respectively; therefore**, 1**, **2**, and **3** were putatively annotated as di-*O*-hexoside, hydroxycitric acid, and citric acid. Metabolite **4** exhibited an absorption band at 270 nm and ions compatible to C_7_H_6_O_5_ (*m*/*z* 169.0137 [M-H]^−^ and 171.0296 [M + H]^+^). From an authentic standard, we confirmed that **4** is the phenol gallic acid, a component of *S. purpurea* seeds [12].

Peaks **5**, **7**, **8**, and **10** showed UV spectra compatible with flavan-3-ols [13], and accurate deprotonated and protonated ions confirmed the molecular formula C_15_H_14_O_7_ and C_15_H_14_O_6_. These components were confirmed by authentic standards as gallocatechin (**5**), epigallocatechin (**7**), catechin (**8**), and epicatechin (**10**). Similarly, compounds **9**, **11-14**, **16-17**, and **19** showed an absorption band at ≈280 nm. These components revealed fragment ions at *m*/*z* 169, 305, and 289 that are consistent with gallic acid, prodelphinidin (gallocatechin/epigallocatechin), and procyanidin (catechin/epicatechin) units. The spectral data were compatible to data reported for O-galloyl prodelphinidin dimer (**9**), *O*-galloyl prodelphinidin-procyanidin (**11**), *O*-galloyl prodelphinidin (**12, 14**), di-*O*-galloyl prodelphinidin dimer (**13**), di-*O*-galloyl prodelphinidin procyanidin (**16**), and *O*-galloyl procyanidin (**17, 19**) [14].

Peak **15** exhibited two absorption bands at 275 and 344 nm in the UV spectrum, similar to coumarin chromophores such as esculetin. Their ions suggested the molecular formula C_10_H_8_O_4_, and the loss of a methyl radical (^•^CH_3_, 15 *u*) confirmed a methoxyl substituent. Thus, compound **15** was annotated as *O*-methyl esculetin [14]. Compound **18** showed a UV spectrum similar to ellagic acid chromophore, in addition to spectral data that suggested **18** was ellagic acid [14], which was confirmed by an authentic standard.

### 3.2. Antioxidant Activity

#### 3.2.1. ABTS and DPPH Radical Scavenging Assay

Direct scavenging assays of the ABTS and DPPH radicals were performed with EBSp and ascorbic acid (AA) and butylated hydroxytoluene (BHT), which were used as standard controls of antioxidant activity (Table 2). In the trial with the ABST radical, the IC_50_ obtained for EBSp was 8 *μ*g.mL^−1^, reaching a maximum inhibition of 94% at 50 *μ*g/mL^−1^, which was not significantly different from the BHT standard. In the direct scavenging assay of the DPPH radical, EBSp behaved similarly to AA, showing a maximum inhibitory activity (91%) at 25 *μ*g.mL^−1^, i.e., more efficient than the standard BHT.

### 3.3. Protection of Proteins against AAPH-Induced Oxidation

The incubation of BSA with the oxidizing agent AAPH promoted BSA oxidation, represented by a decrease in the sharpness of the band and a slight increase in the fragmentation observed below the main band (Figure 1(a)). The graphical representation shows that BSA oxidation increased the band volume by 74% (Figure 1(b)). Furthermore, EBSp reduced the oxidative damage to BSA in a dose-dependent manner beginning at 10 *μ*g.mL^−1^ (15% protection); at a concentration of 100 *μ*g.mL^−1^, EBSp reduced BSA oxidation by 68%.

### 3.4. Protection against DNA Fragmentation Induced by Hydrogen Peroxide and Ultraviolet Radiation

The exposure of plasmid DNA to UV radiation and/or to EBSp (1,000 *μ*g.mL^−1^) was not able to promote DNA fragmentation (Figure 2). The combination of UV radiation and hydrogen peroxide was able to completely fragment the plasmid DNA (Figure 2). Incubation with EBSp is able to significantly protect DNA against fragmentation, with protective effects first observed with 50 *μ*g.mL^−1^ (Figure 2).

### 3.5. Protection against AAPH-Induced Oxidative Hemolysis and Determination of MDA Levels

Erythrocytes incubated with different concentrations of the standard antioxidant AA (5-100 *μ*g.mL^−1^) and EBSp (5-100 *μ*g.mL^−1^) did not undergo hemolysis during the 240 min experimental period (Figure 3(a)). Thus, we evaluated whether the antioxidant properties of EBSp could protect human erythrocytes from AAPH-induced oxidative hemolysis.

The incubation of 50 mM AAPH with human erythrocytes promoted basal hemolysis of 40%. EBSp reduced oxidative hemolysis, promoting reductions of 26, 48, and 65% at concentrations of 10, 50, and 100 *μ*g.mL^−1^, respectively, and was more efficient than the standard AA at low concentrations (Figure 3(b)).

One method used to assess the level of lipid peroxidation that promotes oxidative hemolysis is to measure the MDA content generated. Thus, the level of MDA generated as a result of lipid peroxidation in erythrocytes treated with AAPH was assessed (Figure 3(c)). Incubation with AA reduced MDA levels by 44 and 43% at concentrations of 50 and 100 *μ*g.mL^−1^, respectively. EBSp promoted a significant reduction in the concentration of MDA levels, generating reductions of 37, 36, and 56% at 10, 50, and 100 *μ*g.mL^−1^, respectively.

### 3.6. Hydrogen Peroxide-Induced Oxidative Stress in PBMCs

To investigate the protective effects of EBSp on a second cell model, we used PBMCs incubated with hydrogen peroxide to measure the formation of ROS. PBMCs incubated with hydrogen peroxide (positive control) exhibited a 2-fold increase in ROS levels (Figure 4). When the cells were incubated with hydrogen peroxide and different concentrations of EBSp (5-100 *μ*g.mL^−1^), the ROS levels decreased to the level of the negative control (Figure 4).

### 3.7. Animal Experimentation

#### 3.7.1. Acute Toxicity

After 14 days of oral administration of 2 and 5 g.kg^−1^ EBSp, mice showed no signs of toxicity or mortality, and there were no changes in body mass or food and water intake compared with those for the control group. However, mice in the 2 g.kg^−1^ and 5 g.kg^−1^ groups exhibited increases in the liver of 26 and 22%, increases in leukocytes of 135 and 146%, increases in lymphocytes of 138 and 151%, and reductions in platelet levels of 23 and 28%, respectively (Table 3).

### 3.8. EBSp Activities on Metabolism

Compared to mice fed a standard diet (control group), those fed a high-fat diet (HFD) for 120 days exhibited a 47% increase in body weight (Figure 5(a)). After 60 days of treatment with water (HFD-CT), 30 mg.kg^−1^ simvastatin (HFD-Simv), and 400 mg. kg-^1^ EBSp (HFD-EBSp), the total body mass and the white adipose tissue reserves among mice fed an HFD increased, regardless of treatment (HFD-CT, HFD-Simv, and HFD-EBSp) (Figures 5(a) and 5(b)). Additionally, the caloric intake was similar among all treatments (Figure 5(c)). However, compared with the control mice, mice fed an HFD showed lower water intake (Figure 5(d)).

Compared with the mice fed a standard diet (control group), the obese mice that were treated with water for 60 days (HFD-CT) showed increases of 35, 30, 73, and 188% in the serum levels of cholesterol, triglycerides, glycemia, and ALT, respectively (Table 4). The obese mice treated with simvastatin (HFD-Simv) and EBSp (HDF-EBSp) exhibited 17 and 16% of reduction in cholesterol levels, respectively (Table 4). The serum levels of triglycerides and blood glucose did not differ between the obese groups evaluated, except for a reduction in triglycerides in the HFD-Simv group (Table 4). There were no changes in serum AST levels between mice fed a standard diet and the HFD. The mice fed an HFD that were treated with EBSp (HFD-EBSp) exhibited a significant reduction in serum ALT levels, and mice treated with EBSp had serum levels closest to those of mice fed a standard diet (Table 4).

### 3.9. EBSp Activities against Oxidative Stress

Finally, the levels of MDA in organs were analyzed for signs of oxidative damage from the HFD, and we investigated whether treatment with EBSp could protect the body from damage caused by oxidative stress. The baseline MDA levels in different organs were defined based on the mice fed a standard diet. For the eyes, no significant difference in MDA levels was detected for any treatment. Except for the eyes, the HFD increased MDA levels in all organs evaluated, promoting increases of 84, 157, 224, and 50% in the heart, liver, kidneys, and nervous system, respectively (Figure 6). The group treated with simvastatin (HFD-Simv) exhibited reduced levels of MDA in the heart, liver, and kidneys, levels compared with mice fed with a standard diet. The treatment with simvastatin did not reduce the oxidative damage to the nervous system resulting from the HFD (Figure 6). The group treated with EBSp (HFD-EBSp) showed a reduction in MDA levels in the heart (46%), liver (67%), and kidneys (61%). Furthermore, the ingestion of EBSp prompted a reduction in MDA levels in the nervous system by 72%, the lowest MDA level, even when compared with the baseline levels observed in the group fed with a standard diet (Figure 6).

## 4. Discussion

Oxidative stress conditions produce different levels of damage, i.e., from molecular to systemic. Macromolecules, such as proteins and nucleic acids, can undergo oxidative damage, compromising the catalytic activity and the efficiency of DNA mutation repair. These deleterious effects can cause further changes in cellular components, such as the lipid peroxidation of membrane phospholipids. Thus, cell damage affects tissues, organs, and systems and can trigger the emergence or progression of various diseases, such as obesity, dyslipidemia, diabetes, and cancer [1–4]. Natural compounds with antioxidant properties are able to attenuate oxidative stress, keeping RE levels low and facilitating the prevention and treatment of these diseases [5, 8].

Several phenolic compounds were identified in the stem bark of *S. purpurea*, including some compounds previously described in the species, such as catechin and its derivatives (epigallocatechin, in leaves) [10], gallic acid, kaempferol, and quercetin derivatives (fruit peels) [15]. Other compounds were described for the first time in our study, such as hydroxycitric acid and citric acid. There is a consensus on the contribution of phenolic compounds as important antioxidants; they act through the neutralization of ROS and can modulate the expression of antioxidant enzymes [16–18].

EBSp exhibited broad antioxidant activity, and the synergism of the compounds present in EBSp was comparable to the effects of isolated compounds, such as AA and BHT. The antioxidant action of EBSp is as significant as that observed for fruits of *S. purpurea*, *S. tuberosa*, and *S. dulcis*, for leaves of *S. purpurea*, and *S. dulcis* and for the stem bark of *S. pinnata* [10, 11, 19–21]. The advantage of these properties in *S. purpurea* bark is related to the availability of bark throughout the year, unlike the seasonal availability of leaves and fruits.

REs promote oxidative damage in proteins, DNA, and lipids [22–24]. In this study, we demonstrated that EBSp can protect proteins and DNA from oxidative damage *in vitro*. This protective effect was attributed to the combination of metabolites present in EBSp, as polyphenols and flavonoids are known for such properties [25–27].

*In vitro* protective effects have been observed in complex models, such as cellular models and organisms. Due to their susceptibility to oxidation, erythrocytes have been used as a cell model to investigate damage to biological membranes. Lipid peroxidation promoted by REs leads to the generation of MDA, a marker associated with a variety of diseases [28]. EBSp did not promote erythrocyte hemolysis, suggesting any toxic effects. In addition, EBSp inhibited AAPH-induced lipid peroxidation by reducing the formation of an important end-product, MDA. The reduction in MDA formation in the liver of diabetic animals has also been described for *S. tuberosa* bark extract; this reduction contributed to increased insulin sensitivity and other hepatoprotective effects [29]. We also demonstrated that EBSp protected human peripheral blood mononucleated cells from the accumulation of intracellular ROS induced by H_2_O_2_. A lower ROS generation reduces the deleterious effects of chronic oxidative stress [30, 31], contributing to an increased life expectancy [32].

In the body, oxidative stress occurs in response to an HFD [33, 34]. Increased myocardial lipoperoxidation has been widely described in obese individuals [35, 36], and this factor is associated with a negative prognosis. Therefore, after verification of the absence of mortality and signs of toxicity resulting from the oral administration of high doses of EBSp, which was also evidenced for the stem bark of *S. tuberosa* [37], we investigated the protective effects of EBSp in obese mice to understand the effect of extract consumption on the physiology of these animals.

Obesity induced by the HFD was related to increased body mass, fat deposits, and serum biochemical parameters: elevated blood glucose, cholesterol, and triglyceride levels elevated hepatic ALT levels, and lipid peroxidation in the heart, kidneys, liver, and nervous system. Treatment with EBSp for 60 days prevented lipid peroxidation in the heart, liver, and kidneys and significantly reduced MDA levels in the nervous system. These data suggest that the ingestion of EBSp can help prevent obesity-associated comorbidities described in these tissues, such as hepatic steatosis [30], contributing to an increase in quality of life and life expectancy [32].

The control of serum levels of total cholesterol and triglycerides in the context of obesity is achieved through specific drugs, such as statins. In this study, simvastatin regulated serum levels of total cholesterol and triglycerides in obese mice and reduced lipid peroxidation in the heart, kidneys, and liver. The heart of mice treated with simvastatin exhibited lower MDA levels than those in the control group. However, simvastatin was unable to prevent the lipid peroxidation in the nervous system. The animals treated with EBSp exhibited the same antihypercholesterolemic effects, normalization of the levels of liver damage markers (ALT), and reductions in lipid peroxidation in all organs evaluated, including the central nervous system. These results are supported by the literature, which generally indicates that small amounts of simvastatin cross the blood-brain barrier. High doses of the drug are necessary to reach the nervous system, subsequently producing side effects such as neuropathies [38]. Conversely, catechin, quercetin, and their derivatives, in addition to having direct antioxidant effects, activate signaling pathways that promote the increased availability of antioxidant enzymes [39–41] and have a high ability to cross the blood-brain barrier [42, 43]. Catechin and its derivatives epigallocatechin-3-gallate and (-)-epigallocatechin further promote reductions in cholesterol by inhibiting the synthesis of hydroxy-3-methyl-glutaryl-CoA reductase (HMGR) [44, 45], a mechanism similar to that of simvastatin.

## 5. Conclusion

Several phenolic compounds were identified in EBSp that synergistically contribute to the observed pharmacological, antioxidant, cytoprotective, and antihypercholesterolemic actions. We demonstrated the potential of EBSp in the metabolic control associated with oxidative stress in obese mice, which, in the long term, may prevent the emergence of several comorbidities associated with obesity. Further studies should be conducted to discuss the inclusion of the species *S. purpurea* in the National List of Medicinal Plants of Interest to the Unified Health System (RENISUS, for its acronym in Portuguese), a list created by the Brazilian Ministry of Health to disseminate the use of medicinal plants by Brazilians in the public health system.

## Figures and Tables

**Figure 1:** Protection of proteins against AAPH-induced oxidation. (a) Representative image of 12% SDS-PAGE showing the protective effect of EBSp at increasing concentrations. (b) Graphical representation of the reduction in AAPH-induced BSA oxidation with different concentrations of EBSp (5-100 *μ*g.mL^−1^). The data are presented as the mean ± SEM. The graph was generated using BSA band data from 4 independent gels. ^∗^*P* < 0.05; ^∗∗^*P* < 0.01; and ^∗∗∗^*P* < 0.001 versus EBSp 0 *μ*g.mL^−1^. ^##^*P* < 0.01 and ^###^*P* < 0.001 versus CT (BSA) group.

**Figure 2:** Protection against plasmidial DNA fragmentation induced by H_2_O_2_ and ultraviolet radiation. (a) 1% agarose gel to verify plasmidial DNA integrity and (b) graphical representation of DNA fragmentation after incubation with different concentrations of EBSp (5-100 *μ*g.mL^−1^). The data are presented as the mean ± SEM and were obtained from the analysis of 4 gels. CT: plasmid DNA; CT_UV_: plasmid DNA + ultraviolet radiation; CT_EBSp_: plasmid DNA + ultraviolet radiation + EBSp (1,000 *μ*g.mL^−1^). ^∗∗∗^*P* < 0.001 versus EBSp 0 *μ*g.mL^−1^.

**Figure 3:** Hemolytic activity and protection against AAPH-induced hemolysis. (a) EBSp did not promote hemolysis in human erythrocytes at the concentrations tested. In addition, (b) EBSp inhibited AAPH-induced hemolysis. (c) The levels of MDA generated in the AAPH-induced lipid peroxidation process were significantly reduced when erythrocytes were incubated with EBSp. As a control for antioxidant activity, AA was used at the same concentrations as those used for EBSp. Data are expressed as the mean ± standard error of the mean. ^∗∗^*P* < 0.001 and ^∗∗∗^ compared with the CT group.

**Figure 4:** H_2_O_2_-induced oxidative stress in PBMCs. Mean fluorescence intensity of DCFH-labeled cells (negative control, CT-) incubated with H_2_O_2_ (CT+) and H_2_O_2_ + EBSp (5-100 *μ*g·mL^−1^). EBSp: aqueous extract of the stem bark of *S. purpurea*. The data are presented as the mean ± SEM. ^###^*P* < 0.001 compared to the CT- group and ^∗∗∗^*P* < 0.001 compared to the CT+ group.

**Figure 5:** Anthropometric and metabolic analyses. (a) Evolution of body mass, (b) sum of white adipose tissue deposits, (c) caloric intake, and (d) water intake during obesity induction (0-120 days) and treatment (120-180 days) periods. During the 60 days of treatment (120-180 days), the obese mice received water (HFD-CT), simvastatin (30 mg.kg^−1^ body weight, HFD-Simv), or EBSp (400 mg.kg^−1^ body mass, HFD-EBSp). A group of mice was fed for the same period (180 days) with a standard control diet and water *ad libitum* (control). ^∗∗^*P* < 0.001 compared to the control group.

**Figure 6:** MDA levels in the different organs of mice fed with control or high-fat diet (HFD). Obese mice were treated with water (HFD-CT), simvastatin (HFD-Simv), or EBSp (HFD-EBSp), and after 60 days, oxidative damages in the eyes, heart, liver, kidneys, and nervous system were determined by assessing MDA levels (nmol.mL^−1^). ^∗^*P* < 0.05, ^∗∗^*P* < 0.01, and ^∗∗∗^*P* < 0.001 versus the control group. ^#^*P* < 0.05, ^##^*P* < 0.01, and ^###^*P* < 0.001 versus the HFD-CT group.

**Table 1:** Annotated compounds from aqueous extract of *S. purpurea* stem bark (EBSp) by LC-DAD-MS.

Peak	RT (min)	UV (nm)	MF	Negative (*m*/*z*)		Positive (*m*/*z*)		Compound
				MS [M-H]^−^	MS/MS	MS [M + H]^+^	MS/MS	
1	1.1	—	C_12_H_22_O_11_	341.1089	179	343.1238	—	di-*O*-hexoside
2	1.1	—	C_6_H_8_O_8_	207.0149	189	231.0116^Na^	—	Hydroxycitric acid
3	1.5	—	C_6_H_8_O_7_	191.0196	—	215.0165	—	Citric acid
4	2.4	270	C_7_H_6_O_5_	169.0137	—	171.0296	—	Gallic acid^st^
5	4.2	280	C_15_H_14_O_7_	305.0672	165	307.0818	—	Gallocatechin^st^
6	7.6	—	C_19_H_26_O_13_	461.1322	152	485.1271^Na^	—	Unknown
7	8.6	281	C_15_H_14_O_7_	305.0678	—	307.0810	—	Epigallocatechin^st^
8	9.0	282	C_15_H_14_O_6_	289.0728	203	291.0859	—	Catechin^st^
9	10.0	283	C_37_H_30_O_18_	761.1347	305	763.1511	—	*O*-galloyl prodelphidin dimer
10	12.4	282	C_15_H_14_O_6_	289.0745	—	291.0859	—	Epicatechin^st^
11	12.8	280	C_37_H_30_O_17_	745.1407	—	747.1560	289	*O*-galloyl prodelphidin-procyanidin
12	12.9	274	C_22_H_18_O_11_	457.0814	169	459.0930	307, 289	*O*-galloyl prodelphinidin
13	13.2	278	C_44_H_34_O_22_	913.1587	—	915.1617	457	di-*O*-galloyl prodelphinidin dimer
14	14.5	275	C_22_H_18_O_11_	457.0811	169	459.0918	307, 153	*O*-galloyl prodelphidin
15	15.2	275, 344	C_10_H_8_O_4_	191.0352	—	193.0499	178	*O*-methyl esculetin
16	15.7	280	C_44_H_34_O_21_	897.1513	—	899.1660	459	di-*O*-galloyl prodelphinidin procyanidin
17	17.0	276	C_22_H_18_O_10_	441.0978	169	443.0978	273	*O*-galloyl procyanidin
18	17.6	270, 366	C_14_H_6_O_8_	301.0010	245, 229, 217, 173	303.0130	—	Ellagic acid^st^
19	18.0	276	C_22_H_18_O_10_	441.0847	289, 169	443.0977	291	*O*-galloyl procyanidin

RT: retention time; MF: molecular formula; ^Na^: [M + Na]^+^; ^st^: confirmed by authentic standard.

**Table 2:** ABTS and DPPH scavenging assay for the aqueous extract of the stem bark of *S. purpurea* L. (EBSp) and standard antioxidants.

Sample	ABTS			DPPH		
	IC_50_ [*μ*g.mL^−1^]	Maximum inhibition		IC_50_ [*μ*g.mL^−1^]	Maximum inhibition	
		%	[*μ*g.mL^−1^]		%	[*μ*g.mL^−1^]
AA	4.9 ± 0.30^a^	93	10	4.3 ± 0.20^a^	92	25
BHT	9.0 ± 1.40^a^	98	50	15.2 ± 1.50^b^	80	50
EBSp	8.1 ± 1.20^a^	94	50	7.1 ± 0.70^a^	91	25

AA: ascorbic acid, BHT: butylated hydroxytoluene (BHT), EBSp: aqueous extract of *S. purpurea* stem bark. IC_50_: half maximal inhibitory concentration of EBSp necessary for scavenging ABTS and DPPH. Values are expressed as the mean ± SEM.

**Table 3:** Acute toxicity in organ and hematological parameters of female mice treated with 2 and 5 g of kg^−1^ EBSp orally.

Parameters	Control	2 g.kg^−1^	5 g.kg^−1^
Body mass (%)	100.5 ± 0.5^a^	100.3 ± 0.4^a^	102.7 ± 1.0^a^
Liver (g.100 g^−1^ BW)	4.03 ± 0.07^a^	5.07 ± 0.25^b^	4.96 ± 0.18^b^
Kidney (g.100 g^−1^ BW)	1.12 ± 0.04^a^	1.11 ± 0.06^a^	1.12 ± 0.03^a^
Spleen (g.100 g^−1^ BW)	0.31 ± 0.02^a^	0.32 ± 0.02^a^	0.30 ± 0.02^a^
Heart (g.100 g^−1^ BW)	0.50 ± 0.02^a^	0.51 ± 0.01^a^	0.53 ± 0.01^a^
Lung (g.100 g^−1^ BW)	0.66 ± 0.02^a^	0.72 ± 0.02^a^	0.74 ± 0.07^a^
CNS (g.100 g^−1^ BW)	1.79 ± 0.05^a^	1.92 ± 0.05^a^	1.72 ± 0.07^a^
Erythrocytes (10^6^.*μ*L^−1^)	10.26 ± 0.40^a^	9.68 ± 0.09^a^	9.44 ± 0.11^a^
Hemoglobin (g.dL^−1^)	14.22 ± 0.47^a^	13.82 ± 0.15^a^	13.40 ± 0.23^a^
Hematocrit (%)	56.46 ± 2.51^a^	53.86 ± 0.61^a^	51.54 ± 0.59^a^
MCV (fL)	54.98 ± 0.51^a^	55.62 ± 0.42^a^	54.60 ± 0.31^a^
MCH (pg)	13.86 ± 0.12^a^	14.26 ± 0.11^a^	14.18 ± 0.13^a^
MCHC (%)	25.22 ± 0.30^a^	25.68 ± 0.05^a^	26.00 ± 0.16^a^
RDW-SD (fL)	26.48 ± 0.57^a^	26.12 ± 0.16^a^	25.84 ± 0.40^a^
RDW-CV (%)	19.82 ± 0.40^a^	18.72 ± 0.12^a^	18.70 ± 0.07^a^
Platelet (10^3^.*μ*L^−1^)	919.00 ± 244.00^a^	706.20 ± 34.86^b^	661.00 ± 31.26^b^
Leucocytes (10^3^.*μ*L^−1^)	2.06 ± 0.25^a^	4.83 ± 0.41^b^	5.07 ± 0.23^b^
Neutrophil (%)	0.09 ± 0.03^a^	0.11 ± 0.01^a^	0.08 ± 0.02^a^
Lymphocyte (%)	1.98 ± 0.24^a^	4.71 ± 0.40^b^	4.97 ± 0.24^b^
Monocyte (%)	0.02 ± 0.01^a^	0.01 ± 0.00^a^	0.01 ± 0.00^a^
Eosinophil (%)	0.00 ± 0.00^a^	0.00 ± 0.00^a^	0.00 ± 0.00^a^
Basophil (%)	0.01 ± 0.00^a^	0.00 ± 0.00^a^	0.00 ± 0.00^a^

BW: body weight; CNS: the central nervous system; MCV: mean corpuscular volume; MCH: mean corpuscular hemoglobin; MCHC: mean corpuscular hemoglobin concentration; RDW-SD: red cell distribution width-standard deviation; RDW-CV: red cell distribution width-coefficient of variation. The data are presented as the mean ± standard error of the mean. Different letters indicate significant differences between the groups, with *P* < 0.05.

**Table 4:** Body mass and biochemical parameters of mice fed a standard diet (control-water), high-fat diet (HFD-CT), high-fat diet and simvastatin (HFD-Simv, 30 mg.kg^−1^ MC), or high-fat diet and *S. purpurea* (HFD-EBSp, 400 mg. kg^−1^MC).

Parameters	Control g.100 g^−1^	HFD-CT g.100 g^−1^	HFD-Simv g.100 g^−1^	HFD-EBSp g.100 g^−1^
Cholesterol (mg.dL^−1^)	161.6 ± 1.6^a^	218.4 ± 17.7^b^	181.4 ± 4.6^a^	182.7 ± 3.3^a^
Triglycerides (mg.dL^−1^)	171.1 ± 6.3^a^	221.8 ± 11.5^b^	185.4 ± 3.4^a^	197.0 ± 10.2^ab^
Blood glucose (mg.dL^−1^)	82.5 ± 2.6^a^	143.0 ± 5.6^b^	149.6 ± 5.9^b^	134.3 ± 7.4^b^
AST (U.L^−1^)	82.8 ± 5.6^a^	71.5 ± 6.8^a^	76.3 ± 8.6^a^	62.5 ± 4.5^a^
ALT (U.L^−1^)	24.9 ± 3.3^a^	71.8 ± 8.9^b^	54 ± 10.7^ab^	40.6 ± 8.9^a^

The data are presented as the mean ± standard error of the mean. Different letters indicate significant differences between the groups with *P* < 0.05.

## Data Availability

All data supporting the results are available in the manuscript.

## Supplementary Materials

Supplementary Materials Nineteen compounds were identified in the EBSp by LC-DAD-MS, which were annotated based on their spectral data (UV, MS, and MS/MS) and compared with literature data. Figure S1: base peak chromatograms obtained in positive (a) and negative (b) ionization modes from the aqueous extract of the stem bark of *Spondias purpurea* L. The identified substances are described in Table 1.
